RETRACTED

# Mechanism of Depression through Brain Function Imaging of Depression Patients and Normal People

**DOI:** 10.1155/2022/1125049

**Published:** 2022-01-10

**Authors:** Chaozhi Tang, Yuling Zhang, Zihan Zhai, Xiaofeng Zhu, Chaowei Wang, Ganggang Yang

**Affiliations:** ^1^College of Life Sciences, Henan Normal University, Xinxiang 453007, Henan, China; ^2^Department of Neurology, The First Affiliated Hospital of Xinxiang Medical College, Xinxiang 453100, Henan, China

## Abstract

In recent years, functional magnetic resonance technology has discovered that abnormal connections in different brain regions of the brain may serve as the pathophysiological mechanism of mental illness. Exploring the mechanism of information flow and integration between different brain regions is of great significance for understanding the pathophysiological mechanism of mental illness. This article aims to analyze the mechanism of depression by comparing human brain images of normal people and patients with depression and conduct research. Fluoxetine, a selective 5-HT reuptake inhibitor (SSRI) widely used in clinical practice, can selectively inhibit 5-HT transporter and block the reuptake of 5-HT by the presynaptic membrane. The effect of 5-HT is prolonged and increased, thereby producing antidepressant effects. It has low affinity for adrenergic, histaminergic, and cholinergic receptors and has a weaker effect, resulting in fewer adverse reactions. This paper uses the comparative experiment method and the Welch method and uses the average shortest path length *L* to describe the average value of the shortest path length between two nodes in the network. Attention refers to the ability of a person's mental activity to point and to concentrate on something. Sustained attention means that attention is kept on a certain cognitive object or activity for a certain period of time, which is also called the stability of attention. The research on attention of depression patients generally focuses on continuous attention, and the results obtained show inconsistencies. Most studies have shown that the sustained attention of the depression group is significantly worse than that of the healthy control group. An overview of magnetic resonance imaging technology and an analysis of depression based on resting state were carried out. The key brain areas of the sample core network were scanned, and the ALFF results were analyzed. The data showed that the severity of depression in the depression group was negatively correlated with the ReHo value in the posterior left cerebellum (*P*=0.010). The sense of despair was negatively correlated with the ReHo value in the posterior right cerebellum (*P*=0.013). The diurnal variation was negatively correlated with the ReHo value of the left ring (*P*=0.014). It was positively correlated with the ReHo value of the left ventricle (*P*=0.048). This experiment has better completed the research on the mechanism of depression by analyzing the functional images of patients with depression and normal human brain.

RETRACTED

## 1. Introduction

Inhibition refers to the brain's ability to prevent the input of irrelevant information, suppress the original information or interference information that has nothing to do with the current task, and restrain the activation of inappropriate dominant responses caused by related clues. Research on brain networks related to depression has also become one of the research hotspots in recent years. Some studies use specific tasks to stimulate depression patients and then compare the brain activity of normal controls [1]. It was found that the patient's prefrontal lobe, amygdala, hypothalamus, hippocampus, and other regions had abnormal activities. In addition, studies have also reported that changes in dorsal and frontal lobe activity are positively correlated with depression [2]. The hippocampus is negatively correlated with autocorrelation. The study found that when patients with major depression have negative images related to emotions or text descriptions related to self-processing, the basic nodes of the front and back default pattern network—the posterior cortex and the ventricular prefrontal cortex—are reduced [3, 4].

Depression is one of the most common mental illnesses. According to the latest report of the World Health Organization, depression affects 4.4% of the world's population and causes the most important nonfatal disease burden. Although the basic research of neuropsychiatry has made great progress in recent years, it is still lagging behind to apply the acquired basic research information of depression to the clinic [5]. This is because our understanding of the pathological mechanism of depression is still very good. Limitations, this is also reflected in the heterogeneity of the concept of depression disease and the limited therapeutic effect. Psychiatrists still rely on DSM, ICD, and other systems to diagnose from a symptomatic point of view and lack objective testing tools, such as imaging scans and serological examinations to help diagnose depression, choose treatment, and manage response to treatment. Therefore, the exploration of the pathological mechanism of depression is still a hot and difficult point in current research. Memory is the basis of various human mental activities. Therefore, memory function is very important for normal human mental activities. Memory decline is also one of the common main complaints of patients with depression. There are abundant researches on memory in patients with depression, involving delayed memory of speech, visuospatial memory, working memory, short-term memory, implicit memory, and explicit memory.

RETRACTED

In recent years, many scholars and experts at home and abroad have conducted in-depth thinking and research on this issue. Liu et al. pointed out that delusion is a way for individuals to respond to negative life events. Such people often focus their attention on their own depressive emotions, increase their attention and memory of negative information around them, tend to recall experiences and events related to negative moods, and do not adopt positive attitudes and behaviors. The study did not mention how to solve this problem [6]. Han et al.'s hopelessness theory believes that when individuals experience negative life events, they always view things negatively, thinking that they are incapable and unable to solve problems and often feel helpless and hopeless [7]. Shalini and Sanchita also pointed out those patients with depression have negative biases. Such people always consciously or unconsciously pay attention to negative stimuli in the environment, often have miserable and hopeless thoughts, and often make negative evaluations of themselves and the surrounding environment. This negative bias often affects interpersonal communication and hinders social function [8]. Research by Anusri et al. found that some of the above-mentioned brain areas of the brain have reduced BOLD signal strength when performing some cognitive-related tasks. But his research did not summarize this phenomenon as the concept of negative activation [9]. Stetka mainly used PET technology to extract the BOLD signals of the negatively activated brain regions induced by these tasks and compared them with the signals in the resting state. They found that these brain regions were consistent with the activity level of the whole brain. The brain area is a special activity state in the resting state. However, his research has not confirmed that there is a reliable and stable negative correlation between some active networks and default networks when performing tasks [10]. Perelman compared the activation of the default network of depressed patients and healthy people in the task state and found that the negative activation of the default network increases, that is, patients with depression are more inhibited. However, no specific brain area was pointed out [11]. After Atluri et al. discovered the phenomenon of blood-oxygen-level-dependent signal response, people have new technical means for detecting the brain. But he did not summarize the magnetic resonance imaging technology [12].

RETRACTED

PET is the only new imaging technology that can display the metabolism of biomolecules, receptors, and nerve mediators in the living body. It has been widely used in the diagnosis and differential diagnosis of various diseases, disease judgment, curative effect evaluation, organ function research, and new drug development, etc. The innovations of this article are as follows: (1) It mainly summarizes the research methods, technical methods, and related algorithms used in the article. (2) The average aggregation rate of all nodes in the network is expressed by the algorithm, and the MSC is redefined using the smoothing technique (Welch method). (3) Various parts of the human brain are discussed and analyzed.

## 2. Methods of the Mechanism of Depression through Brain Function Imaging of Depression Patients and Normal People

### 2.1. Data Research Methods of Functional Magnetic Resonance Imaging

In recent years, since the impairment of cognitive function in depression is directly related to the rehabilitation of the social function of patients with depression, research on cognitive impairment in depression has received extensive attention. Cognitive functions include a variety of mental activities such as perception, attention, memory, thinking, executive function, and language comprehension.

Functional magnetic resonance imaging (functional magnetic resonance imaging (fMRI)) is an emerging neuroimaging method, and its principle is to use magnetic resonance imaging to measure the changes in hemodynamics caused by neuronal activity. Due to its noninvasiveness, no radiation exposure problems, and its wider application, fMRI has occupied a place in the field of brain function positioning since the 1990s. It is mainly used to study the brain or spinal cord of humans and animals. The traditional data research method needs to obtain the information under the task state in advance and then compare and analyze it with the subsequent information, but now, the fMRI imaging technology is combined to collect the fMRI data of the subject, in which we can get the difference through different regions of interest (ROI). ROI feature changes information under different time series, so it is no longer necessary to obtain information for comparison in advance, and this data analysis method is based on the fMRI data analysis method [13–15]. At present, there are many methods for fMRI data analysis. According to the degree to which the analysis method depends on the stimulus, the analysis techniques are divided into two categories: one is based on model-driven methods, and the other is based on data-driven methods [16]. The model-driven method is a method based on statistical analysis, and its prerequisite is that the time-to-time images of the pre-brain activity are known. This method is suitable for single functional positioning of the brain, predicting the temporal image of brain activity according to the time of stimulation, and then using the predicted temporal image of brain activity for statistical analysis and positioning [17–19]. A sample image of monitoring using fMRI is shown in Figure 1.

RETRACTED

The condition of cognitive impairment in patients with depression needs to be explored in depth. In addition, there are not many studies on the factors affecting cognitive impairment in patients with depression, mainly focusing on the impact of a single factor on cognitive impairment in patients with depression. The main factors involved are the severity of depression, the first episode, or relapse, whether to take drugs, and the course of the disease. Therefore, it is necessary to conduct further research on the relationship between related factors and cognitive impairment in patients with depression. However, when it comes to the positioning of complex brain functions, data-driven methods are required. The majority of scientific researchers have also proposed many methods of positioning analysis, mainly the following:

1. Principal component analysis (PCA) method [20]: in fMRI technology, the spatial resolution is high, and more ROI areas are often selected during data acquisition, resulting in a larger dimensionality of the fMRI data collected, making the processing process more complicated, so it can be based on some of the ROI data. Contact or functional correlation to compress the data (that is, principal component analysis) retains its main information in the compressed data and then selects features with a higher contribution rate as the signal reflection of fMRI data [21–23]. Depression is a kind of mental illness characterized by significant and lasting depression. It is the main type of mood disorder and one of the common mental disorders. Depression has high morbidity, mortality, and public health costs.
2. Cluster analysis (CA) method [24]: fuzzy cluster analysis technology is an effective method for functional positioning in the research of functional nuclear magnetic resonance data. This method is an exploratory analysis method that can affect the generalization rate of clustering by adjusting the characteristics of the input and then showing the contribution of the input features through the change of the clustering generalization rate [25, 26]. It is an unsupervised analysis method and has good development prospects. Miguel Nicollis calls the brain network a “shared brain-computer interface,” that is, this brain-computer interface is operated by multiple people and applies this technology based on a common goal. For example, physical therapists and doctors can use brain-computer interface technology to take care of or take care of patients in different locations. In the process of clustering analysis of fMRI data, the contribution of clustering features to the cluster generalization rate is used to correlate the functional brain network of the brain and to analyze its positioning. Dopamine is the most abundant catecholamine neurotransmitter in the brain. Dopamine acts as a neurotransmitter to regulate various physiological functions of the central nervous system. Dysregulation of the dopamine system involves Parkinson's disease, schizophrenia, Tourette syndrome, attention deficit hyperactivity syndrome, and pituitary tumors.
3. Independent component analysis (ICA) method: independent component analysis is a type of analysis method used to solve the problem of blind source separation in signal processing [27]. The human brain is a complex system, and different cognitive activities of the brain are often completed by the synergy of multiple brain areas. The fMRI data collected during the experiment has many features that can be extracted but often the data will be mixed with some messy and useless signals. In the process of feature extraction, the interference of these signals is usually removed to find out that can truly reflect the recognition. [28]. The independent component analysis method has a good suppression effect on the influence of noise such as Gaussian. In the process of the experiment, it can accurately eliminate the useless noise and strip the useful nonnoise signal for signal acquisition. Therefore, it is used as a signal analysis method of advanced statistics. Compared with the principal component analysis method, it is more accurate and more widely used. These problems not only bring troubles to patients' daily life, study, and interpersonal relationships but also affect the patients' family life. The onset of depression can be as short as two weeks or more and as long as several years, and most cases have a tendency to recur. It will inevitably bring many problems to the family and society, so timely intervention and treatment of depression are particularly important.

RETRACTED

### 2.2. Resting Function Connection Method

The resting state originally refers to the BOLD signal (fMRI) of people being awake, blindfolded, and relaxed, used to detect abnormalities in brain structure or brain activity. Initially, researchers believed that EEG signals at rest were relatively random and subject to interference. Therefore, in the study of work situations, researchers use the brain activity of participants when they are not working as the basis for the study.

EEG equipment is used to record and amplify changes in the biopotential information inside the brain on the surface of the scalp, reflecting the activity status of different areas of the brain [29]. EEG signal acquisition is a convenient and effective noninvasive way to explore brain activity. The potential changes it reflects are the result of the joint action of many nerve cells in the brain.

The functional connectivity analysis of the resting state EEG mainly consists of three steps as follows: (1) The calculation of the connectivity between different regions of the brain, (2) according to the results of the connectivity, the functional network of the brain and the analysis of related attributes are constructed through the minimum spanning tree, and (3) hierarchical clustering of the minimum spanning tree is different. In this study, the coherence of all 72 electrode EEG signals at each single frequency was calculated by using amplitude squared coherence (MSC). Each element in the coherence matrix represents an estimate of the coherence between the corresponding two electrodes, which indicates the degree of interdependence of different brain regions throughout the brain. Then, a minimum spanning tree (MST) is constructed based on the EEG coherence matrix, and the edges are selected according to the coherence in the process of constructing the minimum spanning tree.  Figure 2 is a process analysis diagram. At present, some studies have explored the relationship between the course of the disease, age, and cognitive impairment in patients with depression, and some studies have explored the influence of factors such as whether to take medication, the degree of depression, and whether it is the first episode. However, related studies mostly use single-factor analysis methods, lacking systematic comprehensive analysis, and the results obtained may be biased.

Alzheimer's disease (AD) is a progressive neurodegenerative disease with insidious onset. Clinically, it is characterized by general dementia such as memory impairment, aphasia, apraxia, agnosia, visual and spatial skills impairment, executive dysfunction, and personality and behavior changes. The etiology is still unknown. Those who have the disease after 65 years old are called Alzheimer's disease.

### 2.3. Introduction to Brain Function Connection

Correlation is the most commonly used linear synchronization method and is defined as follows. Two discrete time series measured at the same time are considered, and then, the cross-correlation function is defined as follows:

(1) $$\begin{array}{c} C_{xy}\left(\tau \right)=\frac{1}{N-t}\sum_{n=1}^{N-\tau }\left(x_{n}-\frac{\bar{x}}{\sigma_{x}}\right)\left(y_{n+t}-\frac{\bar{y}}{\sigma_{y}}\right). \end{array}$$

However, due to the limited size of the collected EEG data signals, in order to accurately estimate the true frequency spectrum, researchers widely use smoothing techniques (Welch's method), so the MSC formula can be expressed as

(2) $$\begin{array}{c} \gamma_{xy}\left(f\right)=\frac{{\left|S_{xy}\left(f\right)\right|}^{2}}{\left|\left\{S_{xx}\left(f\right)\right\}\right|S_{yy}\left(f\right)|}. \end{array}$$

In an undirected network, the aggregation coefficient C can be used to express the aggregation coefficient of *v*2:

(3) $$\begin{array}{c} C_{v2}=\frac{n}{C_{k}^{2}}=\frac{2n}{k\left(k-1\right)}, \end{array}$$

where *k* represents the number of all adjacent nodes of node *v*2, that is, the number of neighbors of node *v*2, and *n* represents the number of edges connected to each other between all adjacent nodes of node v2.

RETRACTED

The average aggregation rate of all nodes in the network can be expressed as

(4) $$\begin{array}{c} C=<C_{i}>. \end{array}$$

When each end of the network has its own weight, the average shortest path length *L* is used to describe the average of the shortest path length between two nodes in the network.

(5) $$\begin{array}{c} L=\frac{1}{N\left(N-1\right)}\sum_{i,j\in V,i\neq j}l_{ij}. \end{array}$$

*d* is defined as the similarity of any two nodes (any two rows in *C*), using Spearman distance calculation.

(6) $$\begin{array}{c} \rho =1-\frac{6\sum d_{i}^{2}}{n^{3}-n}. \end{array}$$

When using statistical analysis methods to study multivariate topics, too many variables will increase the complexity of the topic. People naturally hope that fewer variables will get more information. In many cases, there is a certain correlation between variables. When there is a certain correlation between two variables, it can be explained that the two variables that reflect the information of this subject have a certain overlap. The principal component analysis is to delete the redundant variables (closely related variables) for all the variables originally proposed and establish as few new variables as possible so that these new variables are pairwise unrelated, and these new variables are reflecting keep the original information as much as possible in the information aspect of the subject.

This method of solving problems by adding conditions or restricting requirements is the normalization method. Currently, sLORETA is used more frequently. Through the Monte Carlo comparison and analysis with the MWN and SLF algorithms, it is found that sLORETA has the best effect under different noise intensities and different stimulation depths, and the placement error is the lowest. The calculation process of sLORETA is as follows:

(7) $$\begin{array}{c} \Phi =KJ,\\ F={\left\|\Phi -KJ\right\|}^{2}+\alpha {\left\|J\right\|}^{2},\\ J=Τ\Phi ,\\ T=K^{T}{\left[KK^{T}+\alpha H\right]}^{+}. \end{array}$$

Estimating the standardization of *J* requires estimating its variance.

RETRACTED

In this process, the actual source variance can be seen as

(8) $$\begin{array}{c} S_{j}=I,\;I\in R^{\left(3Nv\right)\times \left(3Nv\right)}. \end{array}$$

In addition, from a Bayesian point of view, the potential difference is due to noise measurement.

(9) $$\begin{array}{c} S_{\Phi }^{\text{noise}}=\alpha H. \end{array}$$

Considering the independence of the actual source activity and the measurement noise, then the potential variance is as follows:

(10) $$\begin{array}{c} S_{j}=TS_{\varphi }T^{T}=T\left(KK^{T}+\alpha H\right)T^{T}=K^{T}{\left[KK^{T}+\alpha H\right]}^{+}K. \end{array}$$

You can get

(11) $$\begin{array}{c} j=TKJ=K^{T}{\left[KK^{T}+\alpha H\right]}^{+}KJ=RJ=S_{J}J, \end{array}$$

in

(12) $$\begin{array}{c} S_{j}=R=K^{T}{\left[KK^{T}+\alpha H\right]}^{+}K. \end{array}$$

When the forecast of each time series is added to the past value of another time series, Granger causality analysis is performed. The specific bivariate autoregressive model is expanded as follows:

(13) $$\begin{array}{c} Y_{t}=\sum_{i=1}^{p}A_{i}X_{\left(t-i\right)}+\sum_{i=1}^{p}B_{i}Y\left(t-i\right)+CZ_{t}+\varepsilon_{t}, \end{array}$$

(14) $$\begin{array}{c} X_{t}=\sum_{i=1}^{p}A_{i}^{\prime }Y_{\left(t-i\right)}+\sum_{i=1}^{p}B_{i}^{\prime }X_{t-i}+C^{\prime }Z_{t}+\varepsilon_{t}^{\prime }. \end{array}$$

Gamma distribution is given by

(15) $$\begin{array}{c} f\left(r\right)=\text{const}\times r^{\left(1-3b\right)/b}\exp\left(-\frac{r}{ab}\right). \end{array}$$

In summary, the introduction of the algorithm is complete, and the experiment is ready to begin.

## 3. Experiments and Analysis of the Mechanism of Depression through Brain Function Imaging Analysis of Depression Patients and Normal People

### 3.1. Preparation before the Experiment

Several patients with major depression were recruited through outpatient clinics. The subjects of the study were all adults (18–60 years old), which matched the individual gender and education level of the normal population in the previous PPI study. They were diagnosed with major depression by an experienced doctor through interviews and using the fourth edition of the Clinical Diagnosis and Statistics Manual of Visceral Diseases. In order to study the relatively stable depression pattern, the following criteria are used to eliminate confounding factors: (1) are you currently receiving or are receiving any antidepressant therapy (antidepressants, psychotherapy, etc.); (2) consolidation or mental illness I; (3) anxiety history of mania and hypomania; (4) under treatment or with neurological diseases; (5) history of head injury and/or drug abuse; and (6) contraindications of magnetic resonance imaging. The severity of depression is assessed by the 17-item Hamilton Depression Inventory (17-HDR) and the second edition of the Beck Depression Inventory (BDI-II). This study strictly followed the “Declaration of Helsinki” and was approved by the Review Committee of the Institute of Ethics of the First Affiliated Hospital of Xinxiang Medical College. In order to protect the rights and interests of the subjects, each person signed and confirmed a written consent form after knowing it. The population data and clinical symptom scores of the subjects are shown in Table 1.

RETRACTED

Cognition is a kind of human mental activity. It refers to the mental process of an individual to recognize and understand things. Cognitive function is composed of multiple cognitive domains, including attention, inhibition, mental operation ability, concept formation and conversion ability, and memory and many other aspects. Cognitive impairment refers to the abnormality of the brain's advanced intelligent processing related to the above-mentioned attention, inhibition, and mental operation abilities, which leads to the damage of attention, inhibition, and mental operation abilities.

Hamilton Depression Scale (HAMD) was compiled by Hamilton in 1960. It is the most commonly used scale in the clinical evaluation of depression. There are 3 versions of this scale, including 17 items, 21 items, and 24 items. This scale is performed by two trained raters to perform a HAMD joint examination on the patient. Generally, speaking and observation are used. After the examination, the two raters separately score independently; scores before and after treatment can evaluate the severity of the disease. Table 1 selects the return on investment previously shown in healthy individual studies and finds the coordinates of the area of interest in the MNI standard. The brain network marker threshold for the independent component analysis is set to *z* > 2.3, and then, all markers for the brain structure of the area of interest and the resting network coordinates of the ICA are recorded, as shown in Table 2.

Although timely intervention can effectively control the disease, most of the patients have repeated attacks, leading to the decline of social function and even suicide in patients with depression. Fifty percent of patients will relapse again within a two-year recovery period, and more than 80% of depression patients will experience more than one stage of depression in their lifetime. The distribution of the region of interest is shown in Figure 3.

RETRACTED

On the other hand, this study found that there is a certain correlation between the right fusiform gyrus of the temporal lobe and the speed of information processing in cognitive function. There is a correlation between the left cerebellum and FAST's cognitive function dimension and total anxiety score. The medial frontal gyrus on the left is correlated with changes in cognitive function dimensions. Two ROIs are defined through a priori theory. These two points represent a brain network that has been fully verified in previous studies. PPI analysis determines the adjustment area of the connectivity between the selected area of interest and the second area of interest and determines the interaction based on the increase or decrease of statistics. For each PPI analysis, we defined two regions of interest (ROI), and each network found this item in the ICA analysis scoreboard. Therefore, PPI analysis will find that the brain area is based on the activity of other brain area networks and the regulation connection of another brain area. This analysis will help you understand the dynamic changes in the brain network connections. The functional connection map of the dorsal, ventral, and posterior insula subregions of the insula is shown in Figure 4.

The overall *t*-test is to test whether the difference between the average of two samples and the population represented by each is significant. The two-population *t*-test is divided into two situations, one is the independent sample *t*-test (there is no correlation between the experimental treatment groups, that is, the independent sample), and the other test is used to test the two groups of unrelated sample subjects obtained difference of the data; the first is the paired sample *t*-test, which is used to test the data obtained by two groups of matched subjects or the difference of the data obtained by the same group of subjects under different conditions. These two situations constitute a sample that is the relevant sample. The key brain areas of the core network are shown in Table 3.

### 3.2. ALFF Results

Recent studies have shown that the acquisition of brain function is both network and local, and the organic combination of the two makes the brain's rich functions. In order to define the local activity of a specific brain area, people put forward the hypothesis that specific signals have local consistency. Based on this, a large number of researchers have used functional magnetic resonance imaging technology to study the brain function activity in the resting state and developed a variety of related characterization methods, such as local consistency ReHo (regional homogeneity). The general information of the three groups of subjects is shown in Table 4.

RETRACTED

It can be seen from Table 4 that the three groups have no significant differences in age and gender composition (*P* > 0.05); there is a significant difference in the number of training years between the depression patient group and the depression-susceptible group (*P* < 0.01). There was no significant difference between the depression sensitivity control group and the normal control group (*P* > 0.05). The fMRI comparison of several groups is shown in Figure 5, and there is no significant difference between the two in the main motor cortex area. But outside the motor cortex, the brain motor function projection network in the normal control group was significantly higher in the lateral insular area than in depression patients (*P* < 0.001). However, some areas of the orbital frontal lobe in depression patients were significantly higher than those in the normal control group (*P* < 0.001).

The correlation between the ReHo value of abnormal brain areas and clinical variables in the depression group is shown in Table 5.

The severity of depression in the depression group was negatively correlated with the ReHo value of the posterior left cerebellum (*P*=0.010). The sense of despair was negatively correlated with the ReHo value of the back of the right cerebellum (*P*=0.013). The diurnal variation is related to the ReHo value of the left ring. It was negatively correlated (*P*=0.014), and positively correlated with the ReHo value of the left ventricle (*P*=0.048).

A sample of subjects with a CUMS stimulating depression phenotype was randomly divided into two groups: a depression group receiving 10 mg/kg fluoxetine solution, once a day, for 21 consecutive days; a depression group and an empty control group receiving the same dose of saline, once a day. Conduct assessment was performed 21 days after the drugs were administered. Fluoxetine should be ready for immediate use. Weight change is shown in Figure 6.

The open-air test is shown in Figure 7.

Figure 7 shows that in the open-air environment, after eight weeks of drug use, it can be found that the subjects moved closer and the degree of depression was deeper. The day experiment in the article is to facilitate the distinction and reduce the content of toxic substances.

Sucrose preference is shown in Figure 8.

It can be seen from Figure 8 that after eight weeks, under the action of the fluoxetine solution, the subjects not only increased their weight significantly but also increased their preference for sucrose, and the degree of depression was higher than that of the normal group.

RETRACTED

The correlation analysis between CPT task indicators and related factors is shown in Figure 9.

According to Figure 9, it can be seen that there is a correlation between the low reporting rate of CPT and the score of the scale (*P* < 0.01), and the course of the disease, whether it is the first episode of these two items and medication, gender, age, and education level. There is a significant correlation (*P* > 0.05). The false-positive rate was related to the time of CPT report, and there was no significant correlation between whether the first episode of the disease occurred and whether the drug was used, gender, gender, age, and education level (*P* > 0.05).

## 4. Discussion of the Mechanism of Depression through Brain Function Imaging of Patients with Depression and Normal People

Current research believes that depression is a mental disorder that involves multiple areas and multiple systems of the brain. At present, a large number of studies using Diffusion Dilation Imaging (DTI) provide a structural basis for the abnormal functional connection of MDD. Compared with the normal control group, the functional connectivity between the DMN and the frontal ventricular blind network in depression patients is reduced. In the cortical border network, the anisotropy score (FA) between the sgACC and the amygdala of adolescent depression patients is reduced. In addition, when depressed patients face terrible faces, the structural activity of the dorsal prefrontal cortex (DLPFC) decreases. All these results indicate that MDD will change in the structural topology of the network.

The functional network of MDD patients has been extensively explored and studied. And a lot of achievements have been made. However, due to the differences in environment, research objects, and analysis methods in the process of experiment and data analysis, different or even opposite results have been found in the research of MDD brain function network. Some research groups have found an increase in brain functional connections in patients with MDD, but some studies have found a decrease in brain functional connections. When building functional connections, most studies usually use thresholds to convert coherence into edges. The choice of threshold has a strong subjective bias, which is also a reason for inconsistent conclusions in different studies that cannot be ignored. In this article, the study uses unbiased methods to build the functional connections of the brain. This method has been used in the research of a variety of mental disorders.

RETRACTED

This research uses the method of functional topology analysis to study the connection between the brain and the functional network. It is verified that the brain function topology obtained has the same pattern as the resting state function network. According to the spatial pattern of the resting brain functional projection network, the functional projection network of the brain was used to compare the topological structure of the functional projection network of the depression group, the depression-susceptible group, and the normal control group and found that there were significant differences in the brain function of the right forehead among the three groups. In some areas of the leaf, the brain function connection of depression-susceptible people is significantly reduced. The motor projection network is also abnormal in the pretreatment depression group, but the abnormal area is located in the lateral insula rather than the main functional area of the motor network. The spatial multivariate regression algorithm is used to map the selected functional network to each thalamus voxel, and the connection distribution of the thalamus voxel and each functional projection network is obtained. Finally, the connection value of the thalamus and each function projection network was compared among the depression group, depression-susceptible people, and the normal control group. The results showed that the connection between the anterior region of the right brain of depression patients and the right subnetwork of CEN was significantly lower than that of the normal control group. It was further found that the functional connection between the entire right thalamus and the right subnetwork of CEN in patients with depression was also significantly lower than that of the right subnetwork of CEN. In the normal control group, the functional connection between the right thalamus and the right subnetwork of CEN was partially restored after treatment, and there was no significant difference from the normal control group. Without correction for multiple comparisons, the connection between the lower part of the brain and the motor network of the depression patients before treatment was significantly lower than that of the normal control group, but there was no significant difference in the connection between the left and right brains and the motor network as a whole.

## 5. Conclusions

The experimental results show that the research on the mechanism of depression through brain function imaging analysis of depression patients and normal humans proposed in this article is more intelligent and scientific in monitoring than other methods of studying the mechanism of depression. Monitoring the cause is also more timely. The article conducted an analysis of depression based on the resting state. The article selected the return on investment previously shown in the study of healthy individuals and found the coordinates of the region of interest in the MNI standard. The author defined two ROIs through a priori theory and performed an fMRI comparative analysis of normal and depressed human brains, and the research on the whole-brain structure network of depression has also been roughly completed. The data showed that the severity of depression in the depression group was negatively correlated with the ReHo value of the left posterior cerebellum, and the sense of despair was negatively correlated with the ReHo value of the right posterior cerebellum. Outside the motor cortex, the brain motor function projection network of the normal control group is significantly higher than that of depression patients in the lateral insular area. The area of the orbital frontal lobe of depression patients was significantly higher than that of the normal control group. The shortcomings of this article are as follows: (1) the data collected by the sample is relatively limited, and the experimental samples can be expanded in future research to obtain the credibility of the research results and (2) the research method in this article only performed fMRI imaging analysis on the human brain but did not control other variables, such as the living habits of the two groups, growth experience, and other variables. This article may be slightly inadequate in rigor. In future research, we can focus on supplementing this piece of content to make the experiment more scientific.

RETRACTED

## Figures and Tables

**Figure 1:** Sample image of monitoring using fMRI.

**Figure 2:** Process analysis. (a) Connectome mapping: using DTI data to build a whole-brain structure network. (b) Topological analysis: comparing the differences in the topological properties of the whole brain through the whole-brain structure network. (c) Fiber tracts analysis: distinguishing the types of fiber damage through the differences in the properties of the three white matter fibers.

**Figure 3:** Distribution of regions of interest.

**Figure 4:** The functional connection map of the dorsal, ventral, and posterior insula subregions of the insula.

**Figure 5:** Comparison of several groups of fMRI.

**Figure 6:** Body weight change.

**Figure 7:** Open-air test.

**Figure 8:** Sucrose preference.

**Figure 9:** Correlation analysis of CPT task indicators and related factors.

**Table 1:** Participant population data and clinical symptom score.

	Depression group	Normal control group	*P* value
Gender (male/female)	7/13	7/13	0.754
Age	41.8 (14.2)	41.6 (13.6)	0.931
Years of education	11.3 (2.6)	10.3 (3.0)	0.305
PANSS		—	—
Positive score	12.9 (5.6)		
Negative score	18.0 (7.0)		
General symptom score	27.8 (5.3)		
Total score	58.7 (12.5)		
HAMD-24		5.3 (1.3)

**Table 2:** Settings and coordinates of interest.

Network name		Brain area	Mini coordinates		
Default network	19	PCC	*X*	*Y*	*Z*
		MPFC	3	−52	26

Executive network on the left	17	LSFG	3	58	6
		LSPL	−33	22	52

Execution network on the right	9	RSFG	−50	−51	50
		RSPL	27	28	52

Highlight the network	13	LIFG	36	−66	48
		LIFG	−48	19	−5

Dorsal attention network	5	RIFG	48	16	−5
		LIPL	−45	−42	56

Auditory network	7	RIPL	48	−39	55
		LSTG	−62	−1	9

Lateral striatum network	20	RSTG	62	−26	16
		LMTG	−50	−65	10

Sports network	1	RMTG	45	−76	10
		LPCG	−48	−7	54
		RPCG	48	−13	54

**Table 3:** Key brain areas of the core network.

Seed point	Brain area	Left and right	Mini coordinates			*T* value
			*x*	*y*	*z*	
Dorsal forebrain insula (to highlight the network)	Ventrolateral prefrontal cortex	Right	33	12	21	12.77
		Left	−36	42	21	10.43
	Temporoparietal junction	Right	63	−33	21	13.87
		Left	−60	−39	21	11.35
	Top leaflet	Right	6	18	30	16.82
		Left	33	−57	39	7.47

Dorsolateral prefrontal cortex (central executive network) posterior cingulate (default network)	Inferior temporal gyrus	Right	−36	−54	36	6.72
		Left	54	−6	−24	7.64
	Angular gyrus	Right	−57	−9	−24	7.82
		Left	51	−51	24	9.61
	Middle back	Right	−42	−75	27	9.9
		Left	24	33	36	9.33
	Medial prefrontal cortex	Right	−27	30	39	7.92
		Left	−3	63	0	8.06
	Para hippocampus	Right	30	−36	−18	6.23
		Left	−33	−42	−18	7.24
	Posterior cerebellum	Left	−9	−60	−48	9.24

**Table 4:** The general information of the three groups of subjects.

	Depression group	Depression-susceptible group	Normal control group	*P*
Age	30.65	31.31	29.33	0.776
Gender	14/9	17/9	8/7	0.748
Education (years)	12.26	16.54	14.53	
HAMD score	29.09	2.27	1.27	

**Table 5:** Correlation between the ReHo value of abnormal brain area and clinical variables in the depression group.

Clinical variables	Brain area	*x*	*y*	*z*	Correlation coefficient (*r*)	*P*
HAMD	Left posterior cerebellum	−3	−75	−30	−0.7597	0.010
Despair	Right posterior cerebellum	3	−81	−30	−0.7655	0.013
Day and night changes	Left cingulate back	−18	−33	30	−0.6106	0.048
Day and night changes	Left thalamus	−3	−9	6	0.7768	0.014

## Data Availability

No data were used to support this study.
